# Food security management in developing countries: Influence of economic factors on their food availability and access

**DOI:** 10.1371/journal.pone.0271696

**Published:** 2022-07-25

**Authors:** Norbert Bozsik, Julieth P. Cubillos T., Bopushev Stalbek, László Vasa, Róbert Magda

**Affiliations:** 1 Institute of Agricultural and Food Economics, Hungarian University of Agriculture and Life Sciences, Gödöllő, Hungary; 2 Doctoral School of Economic and Regional Sciences, Hungarian University of Agriculture and Life Sciences, Gödöllő, Hungary; 3 Faculty of Economics, Hungary and Institute for Foreign Affairs and Trade, Széchenyi István University, Győr, Hungary; 4 Institute of Economics, Hungarian University of Agriculture and Life Sciences, Gödöllő, Hungary; Hungarian University of Agriculture and Life Sciences (MATE), HUNGARY

## Abstract

The research presents an analysis of the food security policy effectiveness on the component of food availability and access in two developing countries, Colombia and Kyrgyzstan, during the period from 2000 to 2018. Determining the state of their food balance trade and the regression analysis for the Food Production Index of the countries, considering four economic indicators. Thus the study attempts to show that policies and strategies have not reached the expected results in terms of reduction of food imports dependency and strengthening of national production and export industry. Furthermore was found that among the economic indicators considered, food inflation, food imports, food exports, and extreme monetary poverty; the last one was the indicator that presented influence on the Food Production Index of both countries, during the period analyzed, showing that access was the main component that defines the food production. The results highlighted the need of integrating food security with the monetary and trade policies of these countries.

## Introduction

Food is an essential component and global concern, directly related to poverty and inequality conditions in a society. The United Nations considers this aspect in the Sustainable Development Goals (SDG) to be achieved by 2030, in the second one, to “end hunger, achieve food security and improve nutrition for all people”. To reach this, one of the strategies is to increase food production by improving soil fertility, using biological resources and advances in genetics [1]

The agricultural production level needs to rise faster than the population growth, without increasing damage to the environment. The main force of development is sustainable intensive farming, which means the more effective utilization of agricultural land and water resources [2]. Thus, emerging concepts such as closing yield gaps, described as the maximum yield potential achievement, considering its agro-ecological conditions, and incorporation of technical and technological efficient strategies [3]; and the integrated farming system, described as an approach to increase food production, reduce environmental footprint through intercropping, and field rotation [4]. Nowadays agriculture raises productivity rapidly, yet it also pays a high price for overconsumption of natural resources and energy use [5], even in some regions is claimed that agricultural food production is related to local natural resources endowment [6].

Therefore, there are concerns of the governments and societies about the food production and the guarantee of access to the population; because it does not involve exclusive the agriculture, since the food sector is influenced also for macroeconomics effects, cultural and social development.

Food security is an important matter for both, researchers and practitioners struggling to provide solutions for supplying sufficient food to the next generations. Numerous remedies and recommendations are given in the literature to bridge the gap between food supply and food demand for the next five decades years [7].

To manage the whole scenario of food, nowadays the food security approach has increased its influence on the nationals’ food policies. For instance, Russia has changed its food policy since 2015 from a food-import dependent country to a food-self-sufficient country [8], whereas China’s long-term Food Policy Plan is to increase agricultural output through improving technology, and land and water management [9]. The importance of the geographical origin of food and the preference for domestic products could also be one of the possible strategies to enhance food safety and sustainability [10–12]

There are policies and strategies that focus mainly on the food production component, however, that is not enough to achieve the end of hunger in developing countries, which have to solve conditions of access, stability, nutrition, distribution, demands, among others. The total amount of food produced should be enough to feed the whole population, nevertheless because of the deficient distribution systems and poverty, about 15% of the world’s population, in developing countries, is undernourished [13], beside the increase of biofuel demand and production [14]. The epidemic crisis caused major disruption to production, investment, and consumer expenditures. This problem is more pronounced in underdeveloped and developing countries [15], which are able to produce the basic food products needed and can influence food security and sustainability [16].

Regarding the analysis of economic components, the impacts of macroeconomic fluctuations on food insecurity have remained scantily explored [17]; some food security studies have analyzed the influence and consequence of economic indicators such as poverty [18, 19], food inflation [20–22], and food balance [6, 23]

Recognizing the importance of the effectiveness of food security policies, and the relevance of economic factors, this study carried out a cross-sectional time-series data (panel data) analysis, to identify, through economic indicators, the progress in the components of food availability and food access, in the food security policy of two developing countries: Kyrgyzstan and Colombia; considering a period from 2000 to 2018, defined due to the availability of indicators data, and the implementation of the food security policy in these countries. Since their policy started to be in force in the same period, Kyrgyzstan in 2007 and Colombia in 2008, both based on the components of food production and access. this lets to analyze the policies results and tendencies in each country [24].

These two countries were selected considering the similarities of their agricultural sectors, such as both concentrate their agricultural commodities in the primary sector, like milk, sugar, vegetables, and fruits products; by 2018 their agriculture share to GDP did not exceed 12% and it had a decreasing trend s an [24]; both countries have considerable challenges on the food insecurity, since the poverty line was 35.7% in Colombia and 20.1% in Kyrgyzstan by 2019 [25]. Besides, they are from regions with a prevalence of undernourished, 7.2% and 8.8%, respectively, by 2018 [26].

The aim of this study is identify the impact of indicators related to macroeconomic context with their consequence at the micro-level [17]. Taking into account that one measure can not capture all dimensions of food security [19], this paper determined the state of the food balance in each country, considering not only exports- imports values, but including the volume tendencies of those trade as well. Besides, it was analyzed the food production index in each country, considering four economic indicators, extreme monetary poverty and food inflation, connected with food access; and food exports and imports, regarding food availability, developing a multiple regression analysis to determine the effects of the four explanatory variables on the food production index of each country. This contributes to determining the most influential economic factor on the foods security management in these developing countries, and to understanding the orientation of the policy’s implementation.

The correlation and multiple regression methods have been widely used to find the relationship between economic status and the food security indicators, applied previously to factors such as food import dependency [27], food balance, dietary data of vegetables and fruits [28], self-sufficiency [29], food price [30], wealth indices and food consumption [31]. Therefore this study considered this statistical analysis (regression model) with the four economic indicators chosen, that have not been studied before in the same model, as is considered in this study.

The analysis of the food security policies’ results in these countries, with these economic indicators, contributes to identifying the most influential economic factor in the food security management of these developing countries, determining, as well, the changes and tendencies in the food balance trade and production index after the implementation of the regulations, arising the questions: Did the food imports dependency reduce after the implementation of food security policy in the countries?, and was food inflation the main influence in the countries’ food production during the period analyzed?.

To develop this, the paper is organized as follows. In the second section, a background of the food security approach was presented, with the state of the countries’ economic indicators, the description of their food security strategies, and their agriculture production. The third section tackles the methods and tools implemented, to identify the balance trade (value and production) of crops and livestock products in both countries, from 2000 to 2018; and the multiple regression analysis. Finally, section four presents the results and discussion, and section five the conclusions of the study.

## Background of the food security approach

“Food security emerged during the 1974 world food crisis as a right to not be undernourished. Neoliberal policies and technocratic conceptions of economic growth and free trade influenced this concept as a development goal” [32]. Since then, there has been an evolution of the concept of food security. By the 1990s the idea of food security had expanded to include not only the access to affordable and nutritious food, but affirmed cultural food preferences as a basic human right” [33]. It enables humans to have physical, economic, and socially acceptable access to a safe and nutritious diet [34].

Food security and “food safety” are subject categories composed far the largest group of articles, whilst subject category “poverty” became considerably smaller. One reason for this may have been the fact that subject category “poverty” was not the focus of research before the world economic crisis [35].

The Committee on World Food Security (CFS), (2009) mentioned that one of the most popular definitions of food security emphasizes its multidimensionality, describing food security as the condition that exists when all people, at all times, have physical, social and economic access to sufficient, safe and nutritious food to meet their dietary needs and food preferences for an active and healthy life [36]. Social capital, and the synergy from interactions of community members, enhance food security status—both directly and indirectly [37]. Thus, Food security gradually and consistently enlarged to involve not only the food availability and food production but also its expansion to ensure explicitly and accessibility of food, simultaneously [38]. The food security approach “prioritizes trade-oriented goods, imports, and intensive agriculture while promoting poverty-alleviation policies” [32].

The importance for governments to develop good management, public policies and guarantee food security in their territories is related to political stability. A food system is made up of the environment, people, institutions, policies, and processes through which food is produced, processed, and brought to the consumer [39], and those who create and enforce food safety regulations need to understand each other’s perspectives better [40]. Developing food supply chains in agriculture could be one of the keys for higher value-added activities and income of the participants along the chains [41]. Those places where hunger is concentrated are also characterized by persistent food insecurity resulting from either food emergencies or man-made crises lasting for several years, those crises may be the result of armed conflict, droughts, floods, the effects of pandemics, among others [42, 43].

Furthermore, adequate management and response to food problems need a contextualized analysis including causal interdependencies, information on climatic aspects, but also on agricultural and socioeconomic indicators [44], which can be useful in the decision-making process of the stakeholders involved. To ensure the countries’ food security, there were strategies such as the stability of prices for necessities, increasing national food production based on smallholder agriculture, and supporting small farmers with seed assistance, labor-intensive programs [45], equipping and infrastructure in rural areas [46], predictable trading systems, by making the international food system more efficient, and trade policies on export and import restrictions [47].

The Existing food security literature includes only few publications that specifically mention co-management as a mechanism through which food security can be enhanced [48]. Food and nutritional security should be operated from intersectoral and interdisciplinary perspectives considering areas as family, local, national and international [33].

Regarding international trade, “this affects food security directly through the impact on food availability, and indirectly through the effects on food accessibility and stability” [49]. Projection of OECD-FAO, (2020) reflects that will remain essential the food security in food-importing countries, and the rural livelihoods in food-exporting countries. Consumers in low-income countries consume the bulk of their calories from vegetable sources, they cannot afford to consume high-priced calories of animal origin [50].

Literature on economic development and policy studies has focused on evaluating specific outcomes from food security policies, nevertheless, is necessary a wider perspective since macroeconomic factors, such as poverty, unemployment and balance trade, play a strong role in the improvement of food security [46].

Recent research claimed that most of the literature is currently focusing on the impact on the price level and volatility, however, it is important to analyze the impact of the trade restriction on food security as well. Trade and trade policies influence the profits of food producers and the food costs for consumers, mainly because of their effect on the world and domestic food prices [49]. The dynamics of food security were not dependent only on the food balance sheets, but on the ability of countries to maintain food consumption through domestic food production, and financing food imports [51].

From 2000 to 2018 Colombia kept a trade surplus on its food balance, except for the years 2012 and 2013 when imports were higher than exports. By 2000 Colombian food imports registered 11.9%, and at the end of the period analyzed, 2018, the food imports were 12.5% [52]. While food exports registered 24.06% in 2000 and 13.6% in 2018.

On its side Kyrgyzstan presented a more fluctuating food balance trade, with a trade deficit in 2007 and the period 2012–2014; this country registered food imports of 14.4% by 2000, moving to 11.1% in 2018. And its food exports in 2000 were around 10.3%, closing in 2018 with 10.6% [52].

However, with this overview is necessary to identify the details of their food balance performance along this time, considering not only the value trade, but the quantity of the production, and analyzing them with the level of domestic food production.

The state of the other economic indicators considered in this research as food inflation showed that starting the period analyzed (2000) was 7% in Colombia and 11% in Kyrgyzstan, finalizing in 2018 with 0.88% to Colombia, and -2.15% to Kyrgyzstan, initially observing a decreasing of food inflation in both that should be studied. Regarding monetary poverty, Colombia registered 23% of its population in 2000, and 15.1 by 2018 [53]. Concerning Kyrgyzstan, monetary poverty declined from 62.6% in 2000 to 22.4% in 2018 [54].

Considering this context and the importance of economic factors in the management of food security, the hypotheses posited to evaluate in this research paper were:

h_1_: “With the implementation of the food security policy there was not a decrease in the food imports amount and dependency, in both countries”
h_2_: “The food access, in terms of food inflation, had a higher effect in the food production index of each country, than the monetary poverty and food balance”

### Context of Colombian food security management

“In Colombia, issues related to poverty are correlated to food security” [33]. According to reports of FAO, at the beginning of 2010, the largest number of people without adequate access to food in Colombia was around 5.7 million people where approximately 57.3% of Colombian households experienced food security, and 42.7% suffered food insecurity [44]. By 2019 the overall national poverty headcount ratio was 35.7% of the population, according to data from World Bank [25], from this 9.5% were vulnerable people in extreme monetary poverty [55].

Colombia has recognized in its constitution of 1991 the right to a balanced diet, which is interpreted by the national legal authorities as the right to food security or timely and permanent access to food to meet nutritional needs [56]. The concept has been related mainly to the agricultural policies, administered by the Ministry of Agriculture and Rural Development, which structures the programs in accordance with the guidelines of the food security policy to encourage food supply and food production.

Since 2008, Colombia developed programs and strategies through the Council of Economic and Social Policy (CONPES) number 113, for the management of food security. It stated that “Food and nutrition security includes sufficient and stable food availability in addition to access and timely, as well as uninterrupted use of the same adequate quantity and quality by all persons under conditions that permit adequate biological use leading to a healthy and active life” [57]. The implementation of this policy is developed by the National Plans for Food Security and Nutrition (PNSAN 2012–2019), which set objectives, strategies and actions to protect the population from hunger and poor nutrition; it seeked to ensure access to food quality in a timely, adequate manner; to ensure that the Colombian population consumes a complete, balanced, enough and adequate diet; with appropriate offer and guarantee access [33].

Furthermore, the PNSAN 2012–2019 proposed the creation of alliances with the private sector to increase competitiveness; according to Roger Merino (2020) with strategies such as financing productive projects with export potential; improving the productivity of small-medium producers, and improving food assistance programs. In practice, the food policies in the country reinforced dependence on imports that damage local economies, single-crop exports, and land-use change for agribusiness expansion over forests and indigenous territories [32].

On its side, the CONPES defined five key components of the Colombian food security and nutritional policy, one of these is availability, which refers to the quantity of food at the national and local level, considering the productive structure, trade system (imports-exports), and political situation. The Access component refers to the ability of people to retrieve adequate and sustainable food supply. The lack of access because of insufficient food amounts, poor delivery, lack of money, and high food costs, are often the causes of food insecurity.

The other three components are Consumption, which means the household food stocks that gather the nutritional needs, diversity, culture, food preferences and education. The biological use component, the way the human body processes the types and quantities of food, and become them in nutrients. The last component is the quality and food safety, refers to food characteristics that make them suitable for human consumption. This component requires the existence of an adequate food chain from production until consumption.

Regarding the economic dimension or perspective of the Colombian food security and nutritional policy, it includes two of the components, Availability (offer or supply of food) and Access (with extreme poverty as an indicator of no access to the minimum type and quantity of food required); this economic dimension will be the emphasis to analyze in this research paper.

The current Colombian Agricultural and Rural Development Policy (2018–2022), focuses on two main aims, on one hand competitiveness, with transformation and production systems, food safety, and investment. On the other hand, rural development is based on employment, infrastructure, social systems and land production [58]. Some of the programs that the Ministry of Agriculture develops in the framework of this policy are “Harvest and sell directly” as a strategy of agriculture marketing, efficient production process, encourage direct trade relationship, and legalize agricultural entrepreneurship [58].

The last “basic food familiar basket” [59] published by the national department of statistics (DANE) in 2017, established the group of basic foods to fulfill nutritional and energy needs. Colombia has 51 basic food products in the groups of cereals; roots and tubers; plantains; vegetables; fruits; meat; fish; and dairy products [60].

By 2020, after twelve years of implementation the CONPES policy and two national plans of food security, the Colombian agriculture sector presented the distribution of its production as shown in Fig 1. The chart presents the share of each crop and livestock products, and can be observed the share of some of the basic food products.

**Fig 1:** Colombian crops and livestock products by 2018 (tonnes), excluded live animals, eggs, hens, other birds in shell. Source: Authors edition based on the FAOSTAT [61].

The crops and livestock products presented in the chart, excluded live animals, eggs, hens, and other birds in shells, to gather specifically production in tonnes. Taking this into account by 2018 the production of 156.088.951 tonnes included 141 agricultural products. The largest production was in the sugar sector with 42.9% (sugar crops primary and sugar cane), followed by milk (9.4%), fruits, oil palm fruit, roots- tubers, and cereals.

The Colombian policy has instruments for the trade defense of agriculture production, such as an early warning system of international trade products and indicators, to provide data for decision-making in the public and private sector. The strategies on food safety focused on participation in international markets. However, in practice, the last agricultural policies, food policies, and the incorporation of 17 trade agreements [62] have reinforced the dependence on imports that affect local economies with the cheapest food, single-crop exports, and land-use change for agribusiness expansion over forests.

Between 2007 to 2018 the cereal import dependency in Colombia kept over 60% and the crops and livestock products import dependency ratio had an increasing trend since 2003, achieving 9.94% in 2018 [61]. Other indicators to identify the current situation and some results of the Colombian Plan of Food Security and Nutrition is the food price inflation, by 2008 in 12.38%, with a decreasing trend until 2016 when drastically raise (12.68%) and low in 2018 until 0.88% [61]. On the other hand, Colombian inflation in 2018 was 2%, according to DANE statistics; with this, it is possible to appreciate the contrast between food inflation and the general inflation in the country [55].

Regarding other international indicators considering in the food security approach, the FAO database [61] registers the Colombian average value of food production to identify the Colombian food availability, and the per capita food supply variability indicator (kcal/capita/day).

### Context of the food security management in Kyrgyzstan

Kyrgyzstan is an agricultural country, and any changes in nature, like natural disasters or climate change, last decades’ draughts and hard winter may lead to undernourishment and food insecurity. Economic and social problems also contribute to malnutrition and food insecurity as the economic gap is essential in Kyrgyzstan, the population of rural regions are less developed than urban ones. In the past 16 years, the level of food security in Kyrgyzstan has only worsened. According to the National Statistical Committee of the Kyrgyz Republic (2019), the population living in poverty is estimated as 22.4%, those who are living in a moderate and severe food insecurity state are 23.9% and the population at the risk of food insecurity condition is 5.1% [63, 64].

The transition from a planned economy into a market economy led to a sharp reduction in subsidies in the mid-90s in the country’s overall economy, and in the agriculture sector particularly. In 1990 and 1995, the GDP crashed by 40 percent, from USD 2.67 billion in 1990 to USD 1.66 billion in 1995 [65]. This trend was followed by a further decline till 2000, such a situation had severe implications for food security in Kyrgyzstan.

This country has been a member of the World Food Program (WFP) since 2011, which has contributed to improving the food security problem, as the programs and advices of The United Nations International Children’s Emergency Fund (UNICEF), who recommended implementing programs on salt iodization and flour fortification, that impacted the health of the population and increase the quality of life. The government adopted the standards of minimum necessary food and calories per person, but the implementation of these standards is low as the level of poverty is high in rural regions [66].

The government identified nine types of basic vital foods products: bread and bakery products, meat and meat products, vegetables and melons, seeds oil, potatoes, milk and dairy products, fruits and berries, sugar, eggs. Above mentioned products are the basic products for assessing the level of food security, taking into account the cultural, historical, climatic characteristics of Kyrgyzstan, and it is set on the Regulation on Monitoring and Food Security Indicators of the Kyrgyz Republic [67]. At the same time, on October 8, 2007, the Regulation on the Food Security Council of the Kyrgyz Republic was adopted.

The causes of the transformational decline in the agrarian economy and a decrease in the level of food security in Kyrgyzstan are considered and given a scientifically based explanation by scientists of the country. The major factors that led to the decline of production in Kyrgyzstan have been associate but not limited to: inflation, lack of financial and other resources, low wages, poor legislative framework, imperfect market structure and infrastructure, irresponsibility of heads of enterprises and government agencies, the prosperity of bribery, corruption, among other [64].

Oruzbaeva (2000) attributes the decline in agricultural production to the ineffective agrarian reform, all the necessary steps of the reform were managed completely by foreign specialists, and as the ineffective result of the reform was an ill-considered choice of strategic directions and methods for their implementation [68]. Contrary, Musaeva (2008) associated the situation to the lack of knowledge and skills of the market mechanism, the price and foreign trade incontinence. Moreover, the change in the material and technical basis of agriculture was affected by the destruction of state farms and collective farms, the formation of family peasant farms through the distribution of land, livestock, and agricultural equipment, that promote manual techniques instead of mechanized agricultural [69].

The ill-conceived agricultural policy leads to unstable development of the agricultural sector and decline of food security. The consequence of this is the destruction of production potential and weak controllability of the agricultural sector. In addition, the marketing and incentive systems for rural producers have developed slowly [70].

Djumabaev (2002) highlighted that one of the main tasks of the Kyrgyz agro-industrial complex is the effective industrialization of agricultural production, which is aimed at providing the population with food, and the processing industries—with raw materials in the volumes necessary for the sustainable development of the food market of the republic. It is necessary to work out a system of economic measurements and legal documents to ensure the country’s food security through domestic production, as well as to create favorable conditions for the life and economic activity of the rural population [71].

According to the Law of the Kyrgyz Republic, the food security is considered to be ensured if the level of the food reserve covers at least 90-days needs of socially vulnerable segments of the population for basic food products. The population with spending below the poverty line is considered as socially vulnerable in Kyrgyzstan (based on the data of the National Statistical Committee of the Kyrgyz Republic in 2018), the population with consumer spending below the poverty line is 22.4% [63].

Despite the growth of basic food products, Kyrgyzstan cannot provide the population with basic food products by its own production (physical inaccessibility), which leads to a high level of food import dependence [72]. The cereal import dependency kept at 16.2% during three years (2016–2018), while the crops and livestock products import dependency was between 4% and 7.89% in the last 5 year [46]. The Kyrgyz production in 2018 was 16.083.438 tonnes, considering specific crops and livestock products in tonnes [61].

Fig 2 let identify the role of the basic vital food products of the countries after 13 years of the regulation on the food security council adoption. Highlighting that cereal, milk, potatoes, roots and vegetable primary (included in the basic vital food) gathered 52.6% of the total production.

**Fig 2:** Kyrgyz crops and livestock products by 2018 (tonnes), excluded live animals, eggs, hen, other birds in shell. Source: Authors edition based on the FAOSTAT [61].

Each region of the Kyrgyz republic is famous with its own product, for instance, the Talas region with beans, Chui—sugar beet, the southern region with tobacco and cotton. Moreover, the country produces dairy products (milk from cows, sheep, goats) and meat products (beef, mutton, horse meat) [73]. Out of all agricultural production livestock production in 2019 was 47.3%, crop production amounted to 50.1%, forestry and services– 2.6% [74]. Some regions have faced land problems and scarcity of water, however, the northern part of the country has better soil.

The food security of Kyrgyzstan gradually fell during the transformation of the national economy, however, there are more reasons that explain the situation and development of food security in the country:

- Unsuccessful reform of the agriculture;
- The gap in the production and technological chain between agriculture and the light and food industries;
- Lack of knowledge and skills of the market mechanism;
- Ill-conceived agricultural policy;
- Reduced government support;
- Lack of modern technology;
- Lack of competitiveness of private farmers.

## Methodology

The analysis of the food security management in each country, was developed with cross-sectional time-series data analysis (panel data), from 2000 to 2018, considering economic indicators to identify characteristics and the impact of the policy and management on the two components, food availability and food access.

The first component of the analysis focuses on the food balance development in each country, to identify the changes in their agriculture production, exports, and imports performance (quantity and trade value), before and after the implementation of the food security policies. The following Table 1 described the indicators and database sources considered in this food balance development.

**Table 1:** Indicators and data sources of food balance analysis.

Indicator	Unit	Source
Crops and livestock products	Tonnes	Calculated base on data from FAOSTAT
Imports quantity: Crops and livestock products	Tonnes	FAOSTAT
Exports quantity: Crops and livestock products	Tonnes	FAOSTAT
Imports value: Crops and livestock products	1000 US$	Calculated base on data from FAOSTAT
Export value: Crops and livestock products	1000 US$	Calculated base on data from FAOSTAT

Source: prepared by authors

The second component is the statistical analysis with the multiple regression method, to identify the effects and model of the four explanatory variables (monetary poverty, food inflation, food imports, and food exports), in the Food Production Index of each country (response variable), presented with details in Table 2. The period analyzed was set from 2000 to 2018, considering the implementation of the food policy in each country and the availability of information.

**Table 2:** Variables and data source for the multiple regression analysis.

Variable	Category	Source	Expected Influence
**Dependent variable**			
Food production index	Food Availability indicator	FAOSTAT	
**Independent (predictor) variables**			
Extreme monetary powerty	Food access indicator	World Bank	negative
Food price inflation	Food access indicator	FAOSTAT	negative
Food exports (% of merchandise exports)	Food availability indicator	World Bank	positive
Food imports (% of merchandise imports)	Food availability indicator	World Bank	negative

Source: prepared by authors

### Definition of indicators for the second component of the methodology

#### Food production Index (2004–2006 = 100)

FAO defines it as the sum of price-weighted quantities of different agricultural commodities produced after deductions of quantities used as seed and feed, and compares a volume of agricultural production in a given year with the base period of reference 2004–2006. Food production index covers food crops that are considered edible and that contain nutrients. Coffee and tea are excluded because, although edible, they have no nutritive value. These indices are given per capita.

To obtain the index number, the aggregate for a given year is divided by the average aggregate of a base period, in this case 2004–2006. National producer prices are expressed as "international commodity prices”, with this is assigned a single price to each commodity (one ton of wheat has the same price in whatever country it was produced).

#### Extreme monetary poverty

According to CEPAL (2018) the poverty line represents a monetary value in which two components are considered: the cost of acquiring a basic food basket and the cost of other goods and services, expressed on the basis of the relationship between total spending and food expenditure [75]. Therefore the calculation of the extreme poverty line corresponds mainly to the value of the basic food basket.

In the case of Colombia the national department of statistics (DANE) builds the basic food basket, selecting products of the food components, guaranteeing the caloric requirement (2100 calories per day) [76]. In case of Kyrgyzstan, like in Colombia, the national statistical committee sets the basic food basket with necessary amount and caloric requirements [63].

#### Food balance trade (imports-exports)

According to the definition of FAO (1996) the food trade means the contribution to food security in different ways. To eliminate the difference between production and consumption, a government imports a lack of basic needed products and exports surplus of produced products in the territory. Thus, a government tries to meet the food needs of the population [77]. However, there are some risks concerning the trade such as increasing the price for importing goods, uncertainty of stability of the world market price, and some political instability.

#### Food price inflation

According to FAOSTAT, Food price Inflation (also known as Consumer Price index) shows the changes of the prices for food over the time that households get for consumption. The International Labour Organization (ILO) is responsible to perform and share the information concerning food price inflation [78].

### Statistical analysis

Considering the previous indicators and the hypothesis h_2_ set, was developed the multiple regression analysis for both countries, with the SPSS program, to determine the influence and effects of the explanatory variables on the food production index, between 2000 to 2018.

#### Multiple regression analysis

This analysis is implemented to predict a dependent variable from two or more independent variables. For this study, there were used as independent variables extreme monetary poverty, food price inflation, food imports, and food exports at once to explain the effects in the dependent variable (Food production index). With multiple regression is possible to forecast the scores on cases for which measurements have not yet been obtained or might be hard to obtain. The regression equation can be used to classify, rate, or rank new cases [78].

This regression includes multiple correlation coefficients such as R and R-squared. R-squared shows what proportion of the variation in the dependent variable is explained by the independent variables. ANOVA sig., in multiple regression helps to assess the overall significance of a model, if P<0,05 the model is significant [79].

### Limitations

There are some limitations to this study to highlighted, regarding the updated data of countries’ indicators in international databases; in some countries do not register the complete information of agriculture sector for all the periods, therefore FAO presented projection due to the lack of official data. On the other side recent indicators on the food security sector (as food insecurity) could not be analyzed since the data registered (from 2014) is not enough to a cross sectional time series analysis. The authors of this research had to do filters of food security indicators with complete reports, for the countries and period of time analyzed in this paper.

It was observed the lack of standard for measuring economic indicators as monetary poverty, since there are regions and countries that implemented their own methodology, the statistics required careful analysis, to compare data between countries; since the calculation of indicators may vary between countries.

## Results and discussion

In this section is presented the two components of the analysis, on one side the tendencies of crops and livestock productions, with the data of exports and imports for both countries; and on the other side, it is detailed the multiple regression running for the response variable, Food Production Index.

### Food balance development

To analyze the performance of exports and imports is important to consider further than the value of the respective balance trade. To analyze the product quantity the traded could give a wider perspective of the imports and exports state in a country. Following is presented the statistics of production, exports and imports of the Crops and livestock products in each country, excluding live animals and eggs, hen, other birds in shell, to enable the calculation of the production in tonnes and their respective value.

#### Food balance of Colombia

The Colombian food security policy sets five lines of action for the economic dimension: stability in the national supply and development of agri-food market; encourage associations and cooperation between companies to boost access to food (free competition); the government priority to design economic and social mechanisms to reduce significant distortions of markets in the food prices; and the international trade policy measures, to guarantee a minimum volume of national production to keep the local food supply.

On his side, Argüello, (2017) claimed that the Colombian export industry did not advance as much as imports, which grew and diversified suppliers, meaning that the number of countries that exported to Colombia increased [80]. In the case of imports, Colombia has both, complementary and substitution relationships with local production, with emphasis on intermediate and capital goods [58].

In the below charts can be appreciated the evolution of Colombian crops and livestock products exports and imports; reflecting on one hand that the internal production is by far higher than the quantity of products exported and imported, guaranteed that most of the national production keeps in the local markets. On the other hand, the quantity of products from imports were higher than exports during all period analyzed; by 2000 with a difference of 1.352.322 tonnes respective the exports quantities, and by 2018 that difference increased to 8.547.953 tonnes.

However, The statistics of the Colombian food trade value, presented a higher value of the food exports during all period, as is observed in Fig 3(b), despite that the amount of exports products were less than imports, these products had a higher economic value; Colombia had a surplus balance on trade value. The values of the food exports and imports were increasing in most of the years, nevertheless is possible to see the reduction in the gap over time; in 2018 the difference value from exports to import was US$3.863.329.000.

**Fig 3:** (a) Colombian production and food balance in tonnes (2000–2018); (b) Colombian food balance value (US$) (2000–2018) tendency. *Source*: Authors edition based on the FAOSTAT [61].

After the implementation of the food security policy (2008), can be observed that there was not large changes in the exports and imports quantities, keeping the growing trend, but even a little stronger for imports. Regarding the total production of crops and livestock products there was not high increase in the period, and in two times were presented reduction, 2009–2010 and 2016–2017, connected with the world economic crisis and in 2016, when there was a national contraction in Colombian exports.

It is important to highlighted that in Latin American countries the crops and livestock production has been influenced to fulfill global food and biofuel market demands [81]. Biofuel and renewable resource policies have boosted the global trade of products as maize, sugarcane, and oil crops [14]. And in the case of Colombia this has increased the participation of the palm oil sector in the national agricultural production. Even the export volume of Colombian palm oil to Europe in 2018 was 252% higher than in 2011, growing faster, than traditional agriculture products such as bananas and coffee, and carrying to the reduction of diversification of agriculture products exported [82].

In practice, the food policies in the country reinforced dependence on imports that damage local economies, single-crop exports, and land-use change for agribusiness expansion over forests and indigenous territories [32]. Reflects that national to enhance competitiveness and productivity of export potential agricultural commodities have not reached the expected results [49].

It is confirmed that there were not a reduction on the imports of food crops and livestock products, showing the same tendencies as the indicator of cereal import dependency presented before. There was a deficit balance regarding trade quantities during all the period analyzed, since, even increasing the tonnes difference between imports and exports and a reduction of the value gap among exports and imports.

Therefore Hypothesis h_1_: “With the implementation of the food security policy there was not a decrease in the food imports amount and dependency, in both countries” is accepted in Colombian case, since there food imports increased in terms of quantity and value.

#### Food balance of Kyrgyzstan

Sun and Zhang have emphasized that the early stages of trade openness among Central Asian (CA) countries have a negative influence on food security; however, beyond a certain level of trade openness, food security status tends to improve; hence, involvement in global markets through international commerce can eventually increase food security in CA countries. The empirical findings further suggest that the other economic and non-economic variables can be key predictors of food security [83].

In Kyrgyzstan, with the advent of the new century, many people migrated to other countries in order to find a new source of income. This greatly affected the country’s agriculture, subsequently it brought a lack of labor force in agricultural sector. Chi et al (2020) reported that the decline of livestock production and crop production is connected with agricultural employment and climatic changes [84]. Subsequently, it brought to the food import dependency.

While in China despite enormous advances in raising food production to maintain national food security over the last decades, China’s food imports have lately increased, which means in some cases government policy is weak towards world uncertainty [9]. This food import in other of the region as Russia has the situation of expensive imported products and devaluation of the rubble have brought to the consumption of cheap substitute products with low quality and decreased purchasing power of the population; the government has achieved food self-sufficiency, but not food security [8].

Kyrgyzstan has a high level of food import dependence, since cannot supply the internal demand of basic food products [72], as can be observed in the below Fig 4, where from 2000 to 2018 the imports were leading the Kyrgyz food balance sheet, with a small decreasing trend since 2009, and the volatile performance of the food exports. In 2018, only three types of basic food products out of nine were achieved by its production: potatoes, vegetables and melons, milk and dairy products. Besides, it is noted from the Fig 4 that there is a big difference considering the measure of food export and food import. The change in exports is not as high from imports in the mass dimension (tonnes), but in value term (US$) there is a significant difference, which can be interpreted the change of the food price over the years.

**Fig 4:** (a) Kyrgyz production and food balance in tonnes (2000–2018); (b) Kyrgyz food balance value (US$) (2000–2018). *Source*: Authors edition based on the FAOSTAT [61].

Most food products such as dairy products, vegetables and melons, fruits are exported mainly to the Eurasian Economic Union (EAEU), mostly to the Russian Federation and Kazakhstan. At the same time, the country depends on imports of some products as wheat, flour, sub-products from meat, poultry, etc. [85].

### Multiple regression for the Food production index

#### Food production index (FPI)

Regarding the indicator Food Production Index, in the period analyzed Colombia had a reduction on the food production, between 2008 and 2010, because of the world economic crisis. After 2010 the trend kept growing, reaching 105,1 in 2009. Coincidentally the food security policy came into force in 2008, but as is observed in the following chart, the positive results on food production started after 2011, even having a faster growth than Kyrgyzstan until 2015.

In the case of Kyrgyzstan, the regulation on food security started in 2007, quite similar to Colombia, however the negative impact of 2008 was less strong in its food production index, and from 2009, it keeps an increasing trend [Fig 5].

**Fig 5:** Food production index of Kyrgyzstan and Colombia, from 2000 to 2018. *Source*: Authors edition based on the Global Economy database [24].

As an indicator of availability, the performance of the food production index for both countries reflected in the above chart lets identify the increase of crop production with nutrients, considering the growth of the population and their food needs, that could be interpreted as a positive result of the policies and food management between 2008 and 2018.

Comparing both countries with the world average index, in the period analyzed, by 2014 the world’s index was 98,2, Colombia had 96,87 and Kyrgyzstan 93.32. After 2016 the index of both countries became higher than the world average (101,2), Colombia (102.65) and Kyrgyzstan (104.58). By 2018 the world’s average was 103.3, Colombia 105.1 and Kyrgyzstan 108.05.

*Multiple regression of FPI in Colombia*. Before the calculation of the regression, was considering the identification of the correlation between the independent variables (extreme monetary poverty, food imports, food exports, and food price inflation).

The result of the correlation, presented in Tables 3 and 4, for the food imports variable, showed that it was not correlated with any other of the three variables. Food exports had correlation with monetary poverty and food inflation, nevertheless, among the correlations presented there were not higher values than 0.6. With this scenario was not affected the collinearity of the regression, since the Tolerance value of the four predictor variables are higher than 0.2 and the Variance Inflation Factors (VIF) are lower than 5, as can be observed in Table 4.

**Table 3:** Model summary and ANOVA.

Model	R	R Square	Adjusted R Square	Std. Error of the estimate
1	.919	.844	.799	4.94234
**ANOVA**		**F**	**Sig**	
**Regression**		18.910	.000^b^	

*Source*: Authors edition based on the SPSS programme [86].

**Table 4:** The results of coefficients for the Colombian multiple regression analysis.

Model	Unstandardized Coefficients		Sig.	Collinearity Statistics	
	B	t		Tolerance	VIF
(Constant)	100.858	9.975	0.000		
Extreme Monetary Poverty	-2.411	-6.467	0.000	0.575	1.740
Food price inflation	0.483	1.214	0.245	0.570	1.754
Food_export	-0.439	-0.755	0.463	0.373	2.684
Food_import	2.136	2.096	0.055	0.737	1.356

*Source*: Authors edition based on the SPSS programme [86].

Regarding the model summary, it presented the correlation between the dependent variable and the independent variables with R: 0.919. the coefficient of determination (R^2^) is 0.84, therefore 84% of the dependent variable is explained by the independent ones. And the standard error of regression was 4.94; this low value indicates that the observations are closer to the fitted line.

In the previous Table 3 also can be observed the significance of the ANOVA, which is lower that 0,05 meaning that this model is significant.

The significance result of the coefficients shows that from the group of the independent variables chosen to analyze the Food Production Index of Colombia between 2000 to 2018, only the Extreme monetary poverty is the predictor variable that is significant, with a coefficient value of -2.411. While the food inflation, food exports and imports were not significant for the Colombian FPI in this scenario.

Thus, the equation of this model is defined as:

$$Y=100.8-2.411*X_{1}\;R^{2}=0.84$$

This model shows a negative relationship between extreme monetary poverty and the Colombian Food production Index, meaning that if the extreme monetary poverty increases to one unit the food production index decreases by an average 2.411 units. Therefore the hypothesis h_2_: “The food access, in terms of food inflation, had a higher effect in the food production index of each country, than the monetary poverty and food balance” is rejected for the Colombian case.

This result that highlighted extreme monetary poverty as the most important economic factor of the food production index of the Country confirm the importance of the food access, in terms of poverty, in the food security management of developing countries, identified as well in countries as Mexico [29], Kenya [30], and Uganda [31].

Regarding the results of not significance for the other independent indicators, in the case of food inflation is important to highlight the heterogeneity of the impacts of inflation on consumption and production patterns. It vary depending of the location, income level, and other household characteristics [21].

The overall impact of food inflation has have been quite different in urban and rural areas. The urban poor are likely to be vulnerable to price surges because their budgets are directly hit by inflated food purchases [22]. While may be benefit to sellers of food, some of whom are poor in rural areas. The inflation of food prices has benefited at least some of the rural farmers, whereas most of the urban poor have been adversely affected [21].

On the other side the trade and trade policies influence the profits of food producers and the food costs for consumers, mainly because of their effect on the world and domestic food prices [49]. The influence of food imports is determined by national factors such as international trade, local demand, agricultural and trade policies, among others.

*Multiple regression of FPI in Kyrgyzstan*. The regression analysis of the Kyrgyz food production index (Y), taking the four independent variables: extreme monetary poverty (X_1_), food imports (% of merchandise imports) (X_2_), food exports (% of merchandise exports) (X_3_), food price inflation (X_4_), presented the following result:

Firstly, the independent variables correlation between each other let identify that food inflation is not correlated with any of the other independent variables, there was found correlation among extreme monetary poverty, food exports and food imports, however this not affect the collinearity statistics. Table 5 shows the fitness of the explanatory variables, because their tolerance values are over 0,10 and VIF values are less than 10. it means there is no multicollinearity. Moreover, the coefficient of determination (R^2^) of the model was calculate in 0.71.

**Table 5:** The results of multiple regression analysis for Kyrgyzstan.

Model	Coefficients (B)	Sig.	Collinearity Statistics	
			Tolerance	VIF
ANOVA		0.001		
(Constant)	117.100	0.000		
Extreme Monetary Poverty	-1.372	0.000	0.241	4.147
Food price inflation	-0.166	0.306	0.850	1.176
Food_export	-0.003	0.430	0.259	3.867
Food_import	-0.010	0.096	0.170	5.887

*Source*: Authors edition based on the SPSS programme [86].

The result of the multiple regression analysis, shows that extreme monetary poverty was the only independent variable that had significance and effects on the food production index of Kyrgyzstan during 2000 to 2018, when is considering in a model with food inflation, food exports and imports.

The significance (P-value) of extreme monetary poverty lower than 0.05 indicates that has influence on the result variable, with a coefficient of -1.345 as it is shown in the Table 5.

It means that there is a negative relationship between the extreme monetary poverty and the food production index of Kyrgyzstan. Thus, the obtained equation for the regression model takes the following form:

$$Y=117.1-1.372*X_{1}\;R^{2}=0.71$$

The determination coefficient of 0.71 means that the extreme monetary poverty influence by 71% in the model. At the same time, if the extreme monetary poverty increases to one unit the food production index decreases by an average 1.372 units. According to the report of WFP (2021), where the extreme monetary poverty decreased from 9.1 in 2006 to 0.5 in 2019 [87] which emphasis the result. Chi et al (2020) study shows that starting from 1995 crop production and livestock production on Kyrgyzstan gradually increased [84]. In 2007, the government developed the regulation on monitoring food security indicators [67]. After the implementation of that regulation, a decrease was found in the poverty line in the country which means the access of population to sufficient food.

Hence, in the case of Kyrgyzstan the hypothesis h_1_ is accepted, since there was not a decrease in food import amount and dependency in Kyrgyzstan. The h_2_ is not accepted while monetary poverty has effect over food production index and food price inflation not.

## Conclusions

The food security policies and regulations are developed in both countries. However, in practice, the policies reinforced food import dependence damaging the internal economy, and neglecting small-farm entrepreneurs, by giving priority to large single-crop producers. Based on the analysis, the effectiveness of the food security management in the countries is faced with various challenges.

In the food balance trade of both countries, was observed that despite the implementation of food security regulation there were not reduction of the food imports dependency. In the case of Colombia the quantity and value of imports grew faster than exports in the period analyzed.

The results of the food security policy, until 2018, had a constant increase in national food production. Nevertheless, did not improve the level of dependence on food imports, to supply the national demand with local production, instead, the level of food import kept a growing trend. Thus, hypothesis h_1_ was confirmed, the strong influence of food imports in these developing countries, keeping the rate in the import dependency indicators, and increasing the quantity and values of the food imports.

Whereas hypothesis h_2_, was rejected since was found that extreme monetary poverty was the variable with influence and effects over the Food Production Index, instead of the food inflation. With the statistical analysis of multiple regression was identified that among the economic indicators analyzed (food inflation, extreme monetary poverty and food exports and imports) is the monetary poverty the most influential factor in the food production index of Colombia and Kyrgyzstan, confirming that food access is the key component in the food security management of developing countries.

This paper tackles two dimensions or components of the food security approach (availability and access), for further research might be suggested to analyze the other two components of food security: utilization and stability, and include social indicators in the assessment of countries.
